# Interactive influences of ecosystem services and socioeconomic factors on watershed eco-compensation standard “popularization” based on natural based solutions

**DOI:** 10.1016/j.heliyon.2022.e12503

**Published:** 2022-12-22

**Authors:** Jian Zhang, Yicheng Fu, Wenqi Peng, Jinyong Zhao, Gensheng Fu

**Affiliations:** a State Key Laboratory of Simulation and Regulation of River Basin Water Cycle, China Institute of Water Resources and Hydropower Research, Beijing 100038, China; b Water Development Planning and Design Co. Ltd., Jinan 250001, China

**Keywords:** Watershed eco-compensation standard, Dynamic equilibrium, Bargaining, Natural based Solutions (NbS), Popularization, Mihe River Basin

## Abstract

Watershed eco-compensation is a policy tool to realize watershed environment improvement and regional economic development. It is important to eliminate the influence of economic differences between upstream & downstream regions and realize the fairness of regional social development based on Natural based Solutions (NbS). At present, lack of clarity in coupling and coordination analysis of ecosystem services & socioeconomic based on NbS could hamper watershed eco-compensation standards “popularization” and reduce the ability to successfully ecological governance. To meet the needs of economic development and ecological service value realization, dynamic equilibrium game research based on multidimensional relationship coordination and a multi-objective optimization solution of economic benefit distribution was carried out. To achieve the bargaining Bayesian/Nash equilibrium of the watershed eco-compensation standard in the game, the existence conditions of the equilibrium solution of the eco-compensation standard based on the mixed equilibrium game implementation process were studied. To carry out the complete information dynamic game, the equilibrium solution of the watershed eco-compensation standard based on the dynamic transfer payment was solved, and the rational analysis of the dynamic Bayesian equilibrium game of bargaining based on the incentive compatibility mechanism was also discussed. Water quantity and quality eco-compensation can ensure balanced development between ecological protection and the social economy in the Mihe River Basin. Combined with the variation law of socioeconomic water intake-utilization standards and the water use value, the city of Shouguang City & Qingzhou City should pay Linqu County 4.78 million US$ and 1.29 million US$ as watershed eco-compensation standards per year based on NbS, respectively. To verify the rationality of the results derived from the economically optimal model, two modes of “bargaining” & “perfect competition”, were used to study the characteristics of the protocols generated by the equilibrium game, and the applicable conditions of the nonzero-sum game solution upstream and downstream of the watershed were also explored. Based on the nonzero-sum processing of the survey results, the current relationship between the input value of eco-compensation and the willingness to pay satisfies v≥c+1/4. Based on the dynamic game & Bayesian equilibrium solution of bargaining, the watershed eco-compensation quota of water quantity & quality is 6.07 million US$, the willingness to pay is 65.63 US$/month. These findings contribute to the quantifying process of bargaining & dynamic equilibrium by transforming “ambiguous” information to achieve sustainable ecosystem service management and develop socioeconomic strategies associated with different compensation features based on NbS, thus helping to inform watershed management.

## 1 Introduction

Watershed eco-compensation is an important means to realize watershed ecological health and sustainable development. Constructing a scientific, reasonable, practical and effective method based on NbS for determining watershed eco-compensation standards has become a research focus in the fields of resources, ecology, the environment, management, the economy and society. A series of research achievements in this area include ecological protection input and ecological benefits around the upstream and downstream regions of the watershed (Bagstad et al., 2013, Li et al., 2017, Zhu et al., 2022a), watershed eco-compensation method determination (Sheng et al., 2020, Shen et al., 2021; Sheng et al., 2022), equilibrium allocation of water resources in catchments (Kosolapova et al., 2017, Fu et al., 2018), determination of contaminant discharge permits for watershed control sections (Guan et al., 2016, Aguilar et al., 2018, Jia et al., 2019, Gao et al., 2019), implementation of sustainable development strategies for watersheds (Fu et al., 2017, Liu and Zhang, 2021, Shang et al., 2022), river and lake health assessment (Nyongesa et al., 2016, Yu and Chen, 2020, Yan et al., 2021), and a systematic, scientific and reasonable computing system was also constructed (Pan et al., 2017, Lu et al., 2021). The existing research results usually consider the meaning and influencing factors of watershed eco-compensation by means of physical value calculation (Yin et al., 2014, Walls and Kuwayama, 2019), measurement of protection costs (Kolinjivadi et al., 2014, Hecken et al., 2015), evaluation of the pollutant governance effect (Tetteh et al., 2006, Zeng et al., 2015, Liu et al., 2021a), regional sustainable development evaluation (Gao et al., 2014, Liang et al., 2017, Zhang et al., 2019a), eco-environmental impact assessment (Liu et al., 2015, Drayson et al., 2015, Ghiasvand et al., 2021) and other relevant mathematical methods. The watershed eco-compensation mechanism according to model calculation, global and local optimization and statistical analysis was studied to realize scientific calculation of the watershed eco-compensation standard (He and Sikor, 2015, Wegner, 2016, Fu et al., 2018). From the influence of the watershed eco-compensation implementation process and the recognition of the complex relationship among different stakeholders, the calculation method of the watershed eco-compensation standard was given based on the results of the equilibrium game calculation under uncertain information. By analyzing the eco-compensation of economics, sociology, law, philosophy connotation, combined with the difficult problem of eco-compensation standard confirmation, based on years of experience in river basin eco-compensation implementation, the calculation of watershed eco-compensation standards based on NbS is urgent. (Chen and Chen, 2019; Jiang et al., 2019a; Mohseni et al., 2021).

Nash's fixed-threat bargaining model (1953) and Roth's Nash equilibrium extension model (1979) provide support for the application of the Nash model in determining watershed eco-compensation standards. Due to the large amount of information contained in the Nash equilibrium model, with the increasing popularity of model application, McDonald and Solow (1981) and Crawford (1982) found that the model had too few quantifiable details, which was not conducive to being widely promoted for empirical or application purposes. To determine the influencing factors in the implementation environment of bargaining, Roth and Malouf (1979) elaborated on the factors represented by the characteristics of the Nash model with the help of experimental results and analyzed the influence of social and psychological factors. Subsequently, Rosenthal and Landau (1979) found that the existence of reputation makes individuals in the population reduce the probability of a bargaining deadlock. On this basis, Rosenthal and Landau (1981) explained the existence of utility uncertainty and the possibility of individuals learning from experience with the help of a self-interested bargaining model. The bargaining game is derived from the free matching of individuals in a group. Social and psychological factors are also key factors affecting the equilibrium of static processes. Gadjov and Pavel (2019) proposed the Nash equilibrium seeking algorithm, which is passive and a game optimization solution using only partial and incomplete information. Persis and Grammatico (2019) took advantage of the passivity of uncertain information games to enrich Nash equilibrium solution methods and construct continuous time gradient functions that combine the equilibrium solution algorithm and distributed mean integral algorithm to carry out dynamic optimization solutions of distributed Nash equilibrium to maximize global fixed incomes. Harsanyi and Selten (1972) and Rubinstein (1982) analyzed how bargaining results were affected by individual behaviors and specific dynamic response characteristics based on an equilibrium game. Machowska et al. (2022) used the principle of state dynamics to construct hyperbolic differential equations for the dynamic solution of partial differential games and used the cumulative return function to carry out the calculation of the double closed-loop Nash equilibrium. When the Nash equilibrium is calculated by a distributed equation, a closed-loop stable game is usually solved by dynamic sharing and gradient dynamics. Since individuals cannot give real-time position changes in each compensation activity and the diversified compensation results are affected by the relative positions of the parties, how to dynamically solve the optimal results based on the equilibrium game model has become the research focus (Wang et al., 2014, Guo and Persis, 2021).

The allocation of ecological resources can be realized by bargaining between the upstream and downstream of the river basin based on NbS. Both sides of the game have some common interests and some opposite views, which is the basis for the balanced solution of the upstream and downstream utility function of the watershed. Based on this, Nash (1953) and Raiffa (1953) proposed modeling the bargaining process by using the extended model and predicting the actual negotiation process in the upper and lower reaches of the basin with the help of the equilibrium solution scheme. A Nash solution is an equilibrium in a one-stage demand game. Scholars have explored the problem of solving multivariate equilibrium games from different angles. Tatarenko and Kamgarpour (2019) used convex inequality constraints to solve equilibrium in multiplayer game processes. Yi and Pavel (2019) carried out an optimization solution of an equilibrium game based on the monotonicity of the coupled group game model. Martinez-Piazuelo et al. (2022) proposed a distributed decision algorithm for optimal solutions in aggregate games with nonlinear aggregate terms and coupled with group game equality constraints. In the case that the upstream and downstream of the watershed implement a common protection plan, the needs of both sides can be met, and then the watershed eco-compensation standard based on NbS can be implemented (Fig. 1).

**Figure 1:** NbS as an umbrella term for watershed eco-compensation related approaches (Cohen-Shacham et al., 2016).

IUCN (2016) defined NbS as protection, sustainable management and restore the ecosystem of the natural or change the action, these actions can be effectively and adaptively to solve the challenges facing the social development, and increase the social welfare and benefits of biodiversity. NbS concepts are used in environmental science and nature conservation to find ways to integrate ecosystem functions to protect ecosystem stability and biodiversity. The process of determining the watershed eco-compensation standard is disturbed by much information and affected by the benefit effect so that the upstream and downstream watersheds cannot reach a consistent agreement. To realize the Nash equilibrium under uncertain informational conditions, scholars have studied the bargaining strategy model from the theoretical level. Crawford (1982) confirmed that the bargaining equilibrium solution can appear in more than one dimension with the help of an efficiency-probability combination. Chatterjee and Ulvila (1982) analyzed multidimensional bargaining problems where participants could determine the optimal compensation strategy with the help of Nash equilibrium solutions. Mg and Mp (2021) analyzed the solution conditions of Bayesian Nash equilibrium pricing. When the benefit value of downstream due to ecological services is greater than the bargaining input of the upstream eco-protection cost, there is no eco-compensation equilibrium solution of the watershed. In contrast, there is a mixed strategy equilibrium in the process of watershed eco-compensation. With the upstream and downstream of the watershed bargain, the price based on the expectation of the ecological restoration subject can be determined by referring to the ecological effect of the watershed.

Based on the connotation and solving process of the Nash equilibrium, the existence conditions of the equilibrium solution of an incomplete information dynamic game, and the feasibility determination of bargaining alliance negotiation, the paper presents a scientific determination method of watershed eco-compensation standards under the influence of multiple information sources, sensitivity of key factors, and economic optimal strategy (Wang et al., 2022; Zhu et al., 2022b). This paper is structured as follows, 1. The introduction elaborates on the theoretical significance of the watershed eco-compensation standard, the development process of the equilibrium game and the Nash equilibrium solution optimization analysis; 2. The materials and methods chapter includes subsections on the (1) Establishment condition of the equilibrium solution of the watershed eco-compensation standard, (2) Equilibrium solution process of the watershed eco-compensation standard, and (3) The bargaining results of the watershed eco-compensation standard; 3. This chapter includes the results and discussion, and 4. The conclusions are reviewed. In view of watershed eco-compensation in the process of parameter implementation, it is not easy to quantify and disturb the calculation method, and the calculation result is not easy to promote. Considering the level of regional social development and ecological protection, the calculation process of the eco-compensation standard was given for the economic optimum and equilibrium, which expands the current watershed eco-compensation standard research methods (Fig. 2). These findings contribute to the quantifying process of bargaining & dynamic equilibrium by transforming “ambiguous” information to ensure recovery of interactive influences of ecosystem services and socioeconomic factors on watershed eco-compensation standard and resilient ecosystems for the long-term benefit of people and nature. We found a disconnection between the implementation preference and the potential value of ecological compensation standards based on NbS. This paper establishes the multivariate equilibrium game model of uncertain information to dynamically determine the watershed eco-compensation standard, determines the rationality of the compensation standard result through bargaining, and explores the watershed eco-compensation standard measurement system based on economic optimization analysis. The innovations are as follows: 1) Coupled watershed eco-compensation standards exist based on equilibrium games, 2) Dynamic Bayesian game equilibrium solution of bargaining optimization is feasible, 3) Bargaining & dynamic equilibrium based on NbS could make eco-compensation standards “popularization”, 4) Necessary condition based on NbS for implementing watershed eco-compensation is v≥c+1/4. These findings contribute to the quantifying process of bargaining & dynamic equilibrium by transforming “ambiguous” information to achieve sustainable ecosystem service management. The research of the thesis has important application value.

**Figure 2:** Flow chart of this study. Based on the analysis of the mechanism of watershed eco-compensation, the influencing factors of compensation standard are analyzed. Based on game theory and equilibrium optimization calculation method, the optimal compensation standard is determined. According to the economic optimization method of compensation standard, the existence condition of compensation standard is given. The study framework of the watershed eco-compensation standard is based on bargaining & dynamic Equilibrium. The dynamic Bayesian game equilibrium solution of bargaining is feasible. The coupling and coordination analysis could make eco-compensation standards “popularization”.

## 2 Materials & methods

### 2.1 Descriptions of study area

The Mihe River is located in the middle of the Shandong Peninsula, and the geographical location is N $118{}^{\circ}36^{\prime }∼119{}^{\circ}8^{\prime }$, E $36{}^{\circ}11^{\prime }∼37{}^{\circ}8^{\prime }$, originating from the west foot of Linqu County and Jiushan town, near the village of Shuishiwu. From south to north, the Mihe River flows through Weifang's Linqu County, Qingzhou City and Shouguang City. In the Coastal Economic & Technological Development Zone, it flows into Bohai Bay. The Mihe River, with a total length of 206 km and a drainage area of 3863 km^2^, is mainly composed of the Shihe River, Danhe River, Shigouhe River and other tributaries (Fig. 3). The terrain of the Mihe River Basin is high in the south and low in the north. To the south of the Jiaoji Railway, there are mostly hills with steep slopes and terrain ratios of 1/50∼1/500. While the north is a plain depression, and the slope is gradual. According to the statistics of precipitation data at Huangshan, Yeyuan Reservoir, Tanjiafang, Hanqiao and other rainfall stations in the basin, the average annual precipitation of the basin is 650.8 mm, and the precipitation from July to September in the flood season accounts for 71.1% of the annual precipitation. The annual average runoff of the Mihe River Basin is 361 million m^3^. According to hydrologic flow data measured by the hydrological stations of the Yeyuan Reservoir and Tanjiafang hydrological stations, the minimum ecological water requirement of the Mihe River Basin is 6.31 million m^3^, which was obtained by using the Tennant method and flow data from 1976 to 2019 (Sun, 2019). The Mihe River Basin is a large sewage discharge river, and its water quality is class V. The water quality of all sections fluctuates at the annual target level (Class IV). Considering that the different sources of water pollutant concentrations exceed the standard, chemical oxygen demand (COD) and ammonia nitrogen (NH_3_-N) were selected as the control indices of point source pollution. Total nitrogen (TN) and total phosphorus (TP) were selected as the control indices of nonpoint source pollution.

**Figure 3:** Location of the Mihe River Basin.

With the improvement of water quality in Shandong Province, there is still a certain gap between the improvement of river water quality and the requirement of surface water function zoning. For the Mihe River, which flows through three cities and counties, it is difficult to clearly define who has invested more and who has invested less in the treatment of river water pollution, as well as has caused more or less pollution. It is difficult to fully mobilize the initiative of the cities and counties in the upper and lower reaches of the river and jointly strengthen the treatment of river water pollution. With the continuous improvement of water quality in Shandong Province, there is still a certain gap between the improvement degree of river water quality and the requirements of water function zone. Mihe River flows through the three cities (counties), it is difficult to make clear who invests more in the treatment of Mihe River and who invests less in the treatment of the Mihe River, and who causes more pollution and who causes less pollution. Therefore, it is difficult to fully arouse the enthusiasm of the cities (counties) to jointly strengthen the treatment of river upstream and downstream. Combining the water distribution and water quality control objectives upstream and downstream of the Mihe River Basin, the computation framework of the eco-compensation standard was given, with the help of the integrity of the watershed water cycle from the aspects of value transfer, social equity and equilibrium game. Therefore, coupling and coordination analysis of ecosystem services & socioeconomic based on NbS could make watershed eco-compensation standards “popularization”.

### 2.2 Data source and data type

The data source, series length and calculation accuracy have important influences on the solution of the watershed eco-compensation standard and optimization of results. The data required for this paper mainly come from data collection and field investigation (Table 1). All foundation data are public and freely available. There are no social ethics and moral problems. Part of the study data comes from the Chinese National Knowledge Infrastructure (CNKI) database and Chinese internet web knowledge.

**Table 1:** Sources of data & information.

### 2.3 Economic valuation coupling & coordination analysis

China is faced with the difficult problem of “dynamic equilibrium and cooperative game” in the implementation of watershed eco-compensation standards. A Nash equilibrium strategy based on economic optimization and transboundary pollution reduction is beneficial to improve the investment level of regional ecological protection and reduce the contaminant stock upstream and downstream. Nash equilibrium calculation process can take into account the service needs and management objectives of different stakeholders. The key of equilibrium calculation is to dynamically realize the optimization objectives that satisfy different users' demand preferences. Fair distribution of ecological goods/public resources is the joint-point of game calculation and Nash dynamic equilibrium calculation of watershed eco-compensation standard. At present, based on the construction of watershed ecological protection compensation standards by natural-based solutions (NbS), evolutionary game theory is used to analyze the evolution trend of strategies of various watershed entities in different situations, and the compensation standards are determined by a simulation model (Unai et al., 2014). Monte Carlo estimation relies on the random distribution function to realize the cooperative work of game alliances. To find the generalized Nash equilibrium of the multivariate game, there is a unique equilibrium in the infinite bargaining game, and dynamic consistency estimation is used to optimize the solution of the decision scheme (Shaked and Sutton, 1984, Wang et al., 2020).

The satisfaction degree of ecological product users and service providers, can be used to popularize the calculation method of watershed eco-compensation standard. To realize the sustainable development of watershed ecosystem services and the socio-economy, the attrition war of ecosystem service value based on the time game is beneficial to realize the cross-regional ecological compensation behavior of watersheds (Maynard Smith, 1974, Lu and He, 2014). Upstream of the watershed, *i* was chosen as the ecological service product $s_{i}\in [0,+\infty )$, while downstream *j* was the expected ecological service product $s_{j}\in [0,+\infty )$. Considering the symmetric information attrition war, when both upstream and downstream of the basin take measures at the same time, the benefit function is:

(1) $$u_{i}(s_{i},s_{j})=\left\{ \begin{array}{cc} -s_{i}\; & s_{j}\geq s_{i}\\ \overset{ˆ}{\theta }-s_{j}\; & s_{j}<s_{i} \end{array}\right.$$

where $\overset{ˆ}{\theta }$ is the expected ecological benefits upstream and downstream of the basin.

Assuming that the cumulative distribution of $\theta_{i}$ is *P* and the density function is *p*, for each $\theta_{i}$, $s_{i}$($\theta_{i}$) should satisfy:

(2) $$s_{i}(\theta_{i})\in \arg\max_{i}\{-s_{i}P[s_{j}(\theta_{j})]\geq s_{i}+\int_{\left\{\theta_{j}|s_{j}(\theta_{j})<s_{i}\right\}}[\theta_{i}-s_{j}(\theta_{j})]p_{j}(\theta_{j})d\theta_{j}\}$$

There is asymmetric equilibrium in this game. That is, in the natural scenario, the upstream tends to choose “implement”, and the downstream tends to choose “withdraw” for watershed eco-compensation. There is a hybrid strategy, symmetric equilibrium in the above games. Each participant determines the feasibility of the eco-compensation implementation strategy according to the distribution function F(s)

(3) $$F(s)=1-\exp(-\frac{s}{\overset{ˆ}{\theta }})$$

The density function of F(s) is given by:

(4) $$f(s)=\frac{1}{\overset{ˆ}{\theta }}\exp(-\frac{s}{\overset{ˆ}{\theta }})$$

The likelihood ratio of F(s) is $ds/\overset{ˆ}{\theta }$. The equilibrium solution exists in the above strategy combination because its expected return is equal to the input cost *ds* ($ds=\overset{ˆ}{\theta }.(ds/\overset{ˆ}{\theta })$). At each moment, if the upstream and downstream of the basin continue to compete for the value of ecological services, the benefits of each participant from this moment will be 0. Therefore, there is no difference in the benefits upstream and downstream of the basin between the implementation and abandonment of eco-compensation strategies.

The hybrid strategy equilibrium of watershed eco-compensation converges to a pure strategy equilibrium. To obtain the continuous distribution sequence with weak convergence to $\overset{ˆ}{\theta }$, it is necessary for watershed upstream and downstream participants to choose a pure strategy. The distribution of equilibrium actions converges to the equilibrium mixed strategy of the corresponding complete information game (Aradillas-López and Rosen, 2022). Considering the symmetric distribution sequence $p^{n}(\cdot )$ on [0,+∞), its cumulative distribution function is $P^{n}(\cdot )$, $P^{n}(0)=0$, and for all ε>0,

(5) $$\lim_{n\to \infty }[P^{n}(\overset{ˆ}{\theta }+\varepsilon )-P^{n}(\overset{ˆ}{\theta }-\varepsilon )]=1$$

Let $s^{n}(\cdot )$ be the symmetric equilibrium strategy corresponding to $p^{n}$, and let $\Phi^{n}$ be the inverse function of $s^{n}$. The expression for $S_{i}(\theta_{i})$ is:

(6) $$s_{i}(\theta_{i})\in \arg\max_{i}\{-s_{i}[1-P_{j}(\Phi_{j}(s_{i}))]+\int_{0}^{s_{i}}(\theta_{i}-s_{j})P_{j}[\Phi_{j}(s_{j})]\Phi_{j}^{\prime }(s_{j})ds_{j}\}$$

By integrating (6), the following is obtained:

(7) $$P^{n}[\Phi^{n}(s)]=1-\exp[-\int_{0}^{s}\frac{1}{\Phi^{n}(b)}db]$$

According to the convergence analysis, the following equation can be obtained:

(8) $$\left\{ \begin{array}{c} \lim_{n\to \infty }P^{n}(\overset{ˆ}{\theta }-\varepsilon )=0\\ P^{n}(\overset{ˆ}{\theta }-\varepsilon )=P^{n}\left[s^{n}(\overset{ˆ}{\theta }-\varepsilon )\right] \end{array}\right.$$

In the same way,

(9) $$\lim_{n\to \infty }s^{n}(\overset{ˆ}{\theta }+\varepsilon )\to \infty$$

When $s^{n}(\overset{ˆ}{\theta }-\varepsilon )<s<s^{n}(\overset{ˆ}{\theta }+\varepsilon )$,

(10) $$P^{n}[\Phi^{n}(s)]=1-\exp[-\int_{0}^{s^{n}(\overset{ˆ}{\theta }-\varepsilon )}\frac{1}{\Phi^{n}(b)}db]\exp[-\int_{s^{n}(\overset{ˆ}{\theta }-\varepsilon )}^{s}\frac{1}{\Phi^{n}(b)}db]=1-[1-P^{n}(\overset{ˆ}{\theta }-\varepsilon )]\exp[-\int_{s^{n}(\overset{ˆ}{\theta }-\varepsilon )}^{s}\frac{1}{\Phi^{n}(b)}db]$$

For all ε>0, then:

(11) $$P^{n}[\Phi^{n}(s)]\to P[\Phi (s)]=1-\exp(-\frac{s}{\overset{ˆ}{\theta }})$$

Comprehensive analysis shows that the equilibrium pure strategy sequence of an incomplete information game converges to the mixed equilibrium strategy of the corresponding complete information game (Aradillas-López, 2011). Therefore, the optimal watershed eco-compensation standard exists in the case of an equilibrium probability distribution.

### 2.4 Quantifying process of dynamic equilibrium methodology

To solve the unique solution of multidimensional action game equilibrium, the payment function model is used to construct the covariance satisfying the game behavior, and the solution of determined parameters under multiple equilibria is carried out (Ht and Tob, 2022, Haque et al., 2022). Chatterjee and Samuelson (1983) considered one of the simplest cases of a bilateral auction, in which a single buyer and a single seller choose whether or not to trade a unit of goods. The input of the cost protection of the seller upstream of the basin is *c*, and the value of the commodity to the buyer downstream of the basin is *v*, where *v* and *c* belong to the interval [0,1]. In the absence of negotiation, both parties choose to bid $b_{1}$ (cost payment upstream of the basin) and $b_{2}$ (willingness to pay downstream of the basin) at the same time, and $b_{1}$ and $b_{2}$ belong to the interval [0,1]. According to the hypothesis of Chatterjee and Samuelson, the transaction price of both auctions is $kb_{1}+(1-k)b_{2}$, where k∈[0,1]. If $b_{1}>b_{2}$, there is no transaction and no currency transfer. If $b_{1}$ is less than or equal to $b_{2}$, price *t* is equal to $(b_{1}+b_{2})/2$. If $b_{1}\leq b_{2}$, the utility in the upper basin is $u_{1}=(b_{1}+b_{2})/(2-c)$; otherwise, it is zero. If $b_{1}\leq b_{2}$, the downstream utility of the basin is $u_{2}=v-(b_{1}+b_{2})/2$ and zero otherwise.

If the upstream and downstream information for eco-compensation is symmetric (i.e., the concept of *v* and *c* shared by the watershed), the above problem is called the Nash demand game (Nash, 1953). To make sense of the problem, the manuscript assumes that v>c; then, there is a continuous pure strategy effective equilibrium in this symmetric information game (Scalzo, 2015). In these equilibria, the upstream and downstream of the basin bid the same, that is, $b_{1}=b_{2}=t\in [c,v]$. Both the upstream and downstream transaction parties of the basin obtained a positive value surplus. If both parties are too “selfish”, and the upstream seller asks more than *t* or the downstream buyer offers less than *t*, the transaction will not take place. At this point, there is an invalid equilibrium in the game, that is, both parties bid at random, the seller asks more than *v* and the buyer offers less than *c*.

The manuscript studied the transaction scenario under asymmetric information. It is assumed that the seller's cost *c* upstream of the basin follows distribution function P_1_ on [0,1], and the buyer's valuation *v* downstream of the basin follows distribution function P_2_ on the same interval. P_1_ and P_2_ have the same characteristics. Chatterjee and Samuelson (1983) proposed a pure strategy equilibrium $s_{1}(\cdot )$ & $s_{2}(\cdot )$ of this game, which is a mapping from interval [0,1] to [0,1]. $F_{1}(\cdot )$ and $F_{2}(\cdot )$ represent the cumulative distribution of bidding in equilibrium (Liu et al., 2017). $F_{1}(b)$ is the probability that the upstream seller of the basin whose cost is *c* will ask no more than *b*

(12) $$F_{1}(b)=P[s_{1}(c)\leq b]$$

Similarly, $F_{2}(b)$ is the probability that the downstream buyer of a basin valued at *v* will bid no more than *b*.

The transfer payment information between the upstream and downstream of the river basin is independent of each other. If the transaction probability is positive, the basin equilibrium offer is an increasing function (Chen et al., 2007). Considering the two types of costs $c^{\prime }$ and $c^{\prime \prime }$, the corresponding strategies of the upstream sellers in the basin are $b_{1}^{\prime }\equiv s_{1}(c^{\prime })$ and $b_{1}^{\prime \prime }\equiv s_{1}(c^{\prime \prime })$, respectively. The optimal strategy requirements of the upstream sellers in the basin are

(13) $$\left\{ \begin{array}{c} \int_{b_{1}^{\prime }}^{1}\left(\frac{b_{1}^{\prime }+b_{2}}{2}-c^{\prime }\right)dF_{2}(b_{2})\geq \int_{b_{1}^{\prime \prime }}^{1}\left(\frac{b_{1}^{\prime \prime }+b_{2}}{2}-c^{\prime \prime }\right)dF_{2}(b_{2})\\ \int_{b_{1}^{\prime \prime }}^{1}\left(\frac{b_{1}^{\prime \prime }+b_{2}}{2}-c^{\prime \prime }\right)dF_{2}(b_{2})\geq \int_{b_{1}^{\prime }}^{1}\left(\frac{b_{1}^{\prime }+b_{2}}{2}-c^{\prime \prime }\right)dF_{2}(b_{2}) \end{array}\right.$$

After comprehensive calculation,

(14) $$(c^{\prime \prime }-c^{\prime })[F_{2}(b_{1}^{\prime \prime })-F_{2}(b_{1}^{\prime })]\geq 0$$

Therefore, if $c^{\prime \prime }\geq c^{\prime }$, then $b_{1}^{\prime \prime }\geq b_{1}^{\prime }$. The manuscript reaches the same conclusion about downstream buyer strategies.

The optimal strategy has increasing, continuous and differentiable characteristics (Mehta et al., 2012). The upstream seller of the basin with a cost of *c* chooses $b_{1}$ to construct:

(15) $$\left\{ \begin{array}{c} \max_{b_{1}}\int_{b_{1}}^{1}\left(\frac{b_{1}+b_{2}}{2}-c\right)dF_{2}(b_{2})\\ \frac{1}{2}\left\{1-F_{2}\left[S_{1}(c)\right]\right\}-\left[s_{1}(c)-c\right]\cdot f_{2}\left[s_{1}(c)\right]=0 \end{array}\right.$$

When cost *c* exceeds the maximum bid from the downstream buyer of the basin, the optimal offer from the upstream seller of the basin is any $s_{1}>{\overset{¯}{s}}_{2}$, and all offers satisfy the seller's first-order condition ($f_{2}[s_{1}(c)]=1-F_{2}[S_{1}(c)]=0$). A similar discussion applies to the downstream buyer's first-order condition. Except when the seller's offer increases to 1, the transaction price only increases by 1/2, and there is no difference between the first-order condition and the monopoly seller's first-order condition (Trofimov and Shalyto, 2013). For the buyer, a similar formula is given as follows:

(16) $$\max_{b_{2}}\int_{0}^{b_{2}}(v-\frac{b_{1}+b_{2}}{2})dF_{1}(b_{1})\;\Rightarrow \;[v-s_{2}(v)]\cdot f_{1}(s_{2}(v))=\frac{1}{2}F_{1}(s_{2}(v))$$

According to the study of Chatterjee and Samuelson (1983), it is assumed that P_1_ and P_2_ are uniformly distributed on [0,1], and the strategy is assumed to be linear.

(17) $$\left\{ \begin{array}{c} s_{1}(c)=\alpha_{1}+\beta_{1}\cdot c\\ s_{2}(v)=\alpha_{2}+\beta_{2}\cdot c \end{array}\right.$$

Based on the above discussion,

(18) $$\left\{ \begin{array}{c} F_{i}(b)=P_{i}\left[s_{i}^{-1}(b)\right]=s_{i}^{-1}(b)=\frac{b-\alpha_{i}}{\beta_{i}}\\ f_{i}(b)=\frac{1}{\beta_{i}} \end{array}\right.$$

Substituting the first-order condition, the following is obtained:

(19) $$\left\{ \begin{array}{c} 2\left[\alpha_{1}+(\beta_{1}-1)c\right]=\left[\beta_{2}-(\alpha_{1}+\beta_{1}\cdot c)+\alpha_{2}\right]/\beta_{2}\\ 2\left[(1-\beta_{2})v-\alpha_{2}\right]/\beta_{1}=(\alpha_{2}+\beta_{2}\cdot v-\alpha_{1})/\beta_{1} \end{array}\right.$$

The above equation holds for all *c* and *v*. The constant terms and the coefficients of *c* and *v* on both sides of the equation should be equal, i.e.,

(20) $$\left\{ \begin{array}{c} 2(\beta_{1}-1)=-\beta_{1}\\ 2(1-\beta_{2})=\beta_{2}\\ 2\alpha_{1}=\beta_{2}-\alpha_{1}+\alpha_{2}\\ -2\alpha_{1}=\alpha_{2}-\alpha_{1} \end{array}\right.\;\Rightarrow \;\left\{ \begin{array}{c} \alpha_{1}=\frac{1}{4}\\ \alpha_{2}=\frac{1}{12}\\ \beta_{1}=\beta_{2}=\frac{2}{3} \end{array}\right.$$

According to the strategy described above, if cost c>3/4 in the upper catchment, its offer (value floor) is 1/4+2c/3 below cost. However, the highest bid $s_{1}(c)$ from the downstream of the basin is also more than 3/4. Therefore, the strategy of the upstream participants will not make them sell the ecological services at a price below the cost. Similarly, when v<1/4, the downstream bid exceeds its value, and the transaction never takes place.

Equilibrium trade occurs if, and only if, $\alpha_{2}+\beta_{2}\cdot v\geq \alpha_{1}+\beta_{1}\cdot c$ or v≥c+1/4. Comparing this condition with the ex post effective trading condition (i.e., trading if and only if v≥c), it can be seen that the trading at equilibrium is too low. Similar to the process of determining symmetric information in game theory, other equilibria exist in this game (De and Machado, 2021). The arbitrary price quote upstream and downstream of the watershed ($b_{1}=1$ & $b_{2}=0$) constitutes an equilibrium. In addition, there is a set of “single price” equilibria on b∈[0,1]. If c≤b, the upstream of the basin offers *b*, and if c>b, it offers 1. If v≥b, the downstream watershed bid *b*. If *v* is less than *b*, bid 0. Since the price is fixed (equal to Tob) when the eco-compensation transaction occurs in the basin, any participant upstream and downstream of the watershed will not change his strategy. Thus, the strategy combination constitutes an equilibrium solution (Ht and Tob, 2022). In addition, Leininger et al. (1989) proved the existence of a single parameter family differentiable symmetric, but nonlinear, equilibrium strategy in this game.

### 2.5 Comprehensive quantitative method for economic bargaining valuation

The upstream, Trader 1, and downstream of the watershed potential buyer, Trader 2, face a single indivisible target, that is the watershed ecological service value, and both parties' utility for money is risk neutral (Lin et al., 2020). The manuscript defines $\overset{˜}{V_{1}}$ as the value of the subject matter to the upstream seller of the basin and denotes $\overset{˜}{V_{2}}$ as the value of the subject matter to the downstream buyer of the watershed. It is assumed that $\overset{˜}{V_{1}}$ and $\overset{˜}{V_{2}}$ are independent random variables, and both follow a uniform distribution on the interval [0,1]. Therefore, the bargaining of the watershed compensation standard is symmetrical and even a transaction.

The thesis assumes that trader *i* is familiar with his valuation at the time of bargaining and treats the other trader's valuation as a random variable. Upstream and downstream traders may communicate with each other, but the trader may not fully disclose the value of the object to him (Ichiishi, 1988). As a direct trading mechanism, the trader simultaneously reports his valuation to a broker, and then determines whether the subject has been transferred from the seller to the buyer, as well as the amount of money the buyer has paid to the seller. The characteristics of the direct transaction mechanism can be expressed by two functions g(⋅,⋅) and x(⋅,⋅). $g(v_{1},v_{2})$ is the probability that the subject is transferred to the downstream buyer, $x(v_{1},v_{2})$ is the expected payment received by the upstream seller, and $v_{1}$ and $v_{2}$ represent the valuation of the seller and buyer, respectively. The valuation reports constitute a Bayesian/Nash equilibrium (Facchinei et al., 2007). Both parties of upstream and downstream transactions in the watershed will truly reflect the true valuation of watershed ecological services. In an incentive compatible mechanism, each trader can maximize his expected utility by realizing his true valuation.

For the Bayesian equilibrium of any bargaining game, there exists an equivalent incentive compatibility direct mechanism, which can produce the same result (Bansal et al., 2022). Given the equilibrium of the bargaining game, the manuscript can construct an equivalent incentive compatibility mechanism: 1) the buyer and seller do not publicly report their valuation; 2) according to these valuations, the actions taken by the trading subject under the given equilibrium strategy are judged; and 3) the possibility of achieving the monetary transfer or the realization of the target is calculated. Refer to Myerson (1979) for more details of the direct mechanism of watershed eco-compensation standards.

According to the direct mechanism of the resultant function (g,x), the function is defined as follows:

(21) $$\left\{ \begin{array}{c} {\overset{¯}{x}}_{1}(v_{1})=\int_{0}^{1}x(v_{1},t_{2})dt_{2}\\ {\overset{¯}{x}}_{2}(v_{2})=\int_{0}^{1}x(t_{1},v_{2})dt_{1}\\ {\overset{¯}{g}}_{1}(v_{1})=\int_{0}^{1}g(v_{1},t_{2})dt_{2}\\ {\overset{¯}{g}}_{2}(v_{2})=\int_{0}^{1}g(t_{1},v_{2})dt_{1} \end{array}\right.\Rightarrow \left\{ \begin{array}{c} U_{1}(v_{1},g,x)={\overset{¯}{x}}_{1}(v_{1})-v_{1}\cdot {\overset{¯}{g}}_{1}(v_{1})\\ U_{2}(v_{2},g,x)=v_{2}\cdot {\overset{¯}{g}}_{2}(v_{2})-{\overset{¯}{x}}_{2}(v_{2}) \end{array}\right.$$

where $U_{1}(v_{1},p,x)$ represents the expected profit or benefit obtained from the transaction when the upstream seller's valuation is $v_{1}$; ${\overset{¯}{x}}_{1}(v_{1})$ is the expected revenue upstream of the basin; ${\overset{¯}{g}}_{1}(v_{1})$ is the probability of losing targets upstream of the basin; $U_{2}(v_{2},g,x)$ is the expected benefit of the downstream buyer from the transaction; ${\overset{¯}{x}}_{2}(v_{2})$ is the expected payment of the downstream buyer of the basin; and ${\overset{¯}{g}}_{2}(v_{2})$ is the probability of the downstream buyer of the basin getting the subject matter.

(g,x) is assumed to be excitation compatible if and only if for every $v_{1}$, $v_{2}$, $t_{1}$ and $t_{2}$ between 0 and 1. There are:

(22) $$\left\{ \begin{array}{c} U_{1}(v_{1},g,x)\geq {\overset{¯}{x}}_{1}(t_{1})-v_{1}\cdot {\overset{¯}{g}}_{1}(t_{1})\\ U_{2}(v_{2},g,x)=v_{2}\cdot {\overset{¯}{g}}_{2}(t_{2})-{\overset{¯}{x}}_{2}(t_{2}) \end{array}\right.$$

The mechanism (g,x) is individually rational (Ck et al., 2021). If and only if any valuation is given, the upstream and downstream of the basin obtain a nonnegative expected return from the transaction, i.e., for each $v_{1}$ & $v_{2}$ between 0 and 1, there are:

(23) $$\left\{ \begin{array}{c} U_{1}(v_{1},g,x)\geq 0\\ U_{2}(v_{2},g,x)\geq 0 \end{array}\right.$$

When the upstream and downstream of the river basin voluntarily entered into the bargaining procedure for the ecological compensation standard, they knew its evaluation. Thus, the feasible mechanism is individually rational (Haimanko, 2021). A mechanism works, if and only if, it is individually rational and incentive compatible. No one wants to facilitate transactions that become worse after the fact. For each $v_{1}$ and $v_{2}$, there are:

(24) $$\left\{ \begin{array}{c} x(v_{1},v_{2})-v_{1}\cdot g(v_{1},v_{2})\geq 0\\ v_{2}\cdot g(v_{1},v_{2})-x(v_{1},v_{2})\geq 0 \end{array}\right.$$

If (1, *g*, *x*) satisfies the above equation, then:

(25) $$\left\{ \begin{array}{c} U_{1}(1,g,x)=0\\ U_{2}(0,g,x)=0 \end{array}\right.$$

The mixed strategy Nash equilibrium exists in every normal game (Fu, 2021). If ${\overset{˜}{V}}_{1}=1$, then the upstream seller is not expected to benefit from the ecological services transaction because he knows that the downstream buyer has a lower valuation. Similarly, if ${\overset{˜}{V}}_{2}=0$, then the downstream buyer in the basin is not expected to benefit from the transaction. Therefore, if the feasible mechanism (g,x) is normative, then $U_{1}(1,g,x)=U_{2}(0,g,x)$ (Lu, 2009).

At this point, for any incentive compatible mechanism (g,x), given the function [0,1]×[0,1]→[0,1], then:

(26) $$\left\{ \begin{array}{c} 0\leq \int_{0}^{1}\int_{0}^{1}(v_{2}-v_{1}-0.5)\cdot g(v_{1},v_{2})dv_{1}dv_{2}\\ U_{1}(1,g,x)+U_{2}(0,g,x)=2\int_{0}^{1}\int_{0}^{1}(v_{2}-v_{1}-0.5)\cdot g(v_{1},v_{2})dv_{1}dv_{2} \end{array}\right.$$

When ${\overset{¯}{g}}_{1}(\cdot )$ is a weakly decreasing function and ${\overset{¯}{g}}_{2}(\cdot )$ is a weakly increasing function:

(27) $$\left\{ \begin{array}{c} U_{1}(v_{1},g,x)=U_{1}(1,g,x)+\int_{0}^{1}{\overset{¯}{g}}_{1}(s_{1})ds_{1}\\ U_{2}(v_{2},g,x)=U_{2}(0,g,x)+\int_{0}^{1}{\overset{¯}{g}}_{2}(s_{2})ds_{2} \end{array}\right.$$

According to the research results of Myerson and Satterthwaite (1983), it can be obtained that:

(28) $$\int_{0}^{1}\int_{0}^{v_{2}}(v_{2}-v_{1}-\frac{1}{3})dv_{1}dv_{2}=0$$

Given ${\overset{˜}{V}}_{2}\geq {\overset{˜}{V}}_{1}$ (everyone upstream and downstream of the basin can benefit from the transaction), the ${\overset{˜}{V}}_{2}-{\overset{˜}{V}}_{1}$ expected value is equal to 1/3. For any feasible mechanism, the ${\overset{˜}{V}}_{2}-{\overset{˜}{V}}_{1}$ expected value is at least 1/2 if the transaction actually happens.

For balanced transactions with symmetric information, each ${\overset{˜}{V}}_{1}$ & ${\overset{˜}{V}}_{2}$ are independent events. The downstream buyer and the upstream seller have at most one opportunity to exchange information with each other (to avoid repeated game), and the ${\overset{˜}{V}}_{2}-{\overset{˜}{V}}_{1}$ average value should be close to 1/2. This prediction holds regardless of how social habits and watershed characteristics affect the negotiation process (Msm et al., 2021). Since no one wants to make a losing deal, the upstream and downstream reaches of the basin trade with the objective of achieving some kind of Bayesian/Nash equilibrium in the bargaining game.

Stated in a geometric sense (Fig. 4(a)), the dotted line represents the set of points $v_{2}=v_{1}+1/2$. Draw any increasing curve on the unit square, such that the center of gravity of the area above the curve falls on or above the dotted line; then, there is some feasible mechanism for the transaction to occur if and only if $\left({\overset{˜}{V}}_{1},{\overset{˜}{V}}_{2}\right)$ is above the curve. For a canonical mechanism, the center of gravity must fall on the dotted line.

**Figure 4:** To realize the contribution of eco-compensation to sustainable watershed development through NbS & ecosystem approaches. The change of watershed's main function will inevitably lead to the change of watershed's ecological service value. Therefore, based on the analysis framework of watershed value transfer, a tradeoff model of ecological protection input and economic value was established to analyze the relationship between ecological protection and economic development. Dramatic growth in water resource utilization efficiency over two decades. The mainstay of watershed eco-compensation in China is related to the large-scale water resources management and water quality improvement programs.

## 3 Results analysis

### 3.1 Interactive coupling analysis between physical properties & ecosystem service

#### 3.1.1 Water release calculation based on ecosystem services & values

With the rapid development of the economy and the rapid increase in population, water consumption in the Mihe River Basin has increased sharply, and the contradiction between upstream and downstream water consumption is evident. To rationally utilize water resources in the Mihe River Basin and improve water resource utilization efficiency, entropy value theory was used to realize system equilibrium and stability from the perspective of the maximum coordination degree of the three-dimensional system of socioeconomic development level, ecological environment succession and the change water resource quality. As a dissipative structure, the intake and drainage relationship between the water resources system, the eco-economic system and the natural environment, as well as the supply-demand and invocation relationship between the water resources system and eco-economic system, conform to the characteristics of dynamic equilibrium, circulation and regeneration (Sn et al., 2021, Xu et al., 2022). To ensure the normal and sustainable exchange of matter, energy and information between the water resources system of the Mihe River Basin and the external natural environment and eco-economic system, the vector projection analysis relation of interaction between the systems is given.

(29) $$\max(S)=\int_{t_{1}}^{t_{2}}F(Es,Ee,Wr)dt\begin{array}{cc} \; & S>0 \end{array}$$

$$\left\{ \begin{array}{c} Es=\int_{t_{1}}^{t_{2}}F(Ee,Wr)dt\\ Ee=\int_{t_{1}}^{t_{2}}F(Es,Wr)dt\\ Wr=\int_{t_{1}}^{t_{2}}F(Ee,Wr)dt>0 \end{array}\right.$$

where *S* is the coordination degree between systems, *Es* is the human economic and social system and its closely related artificial environment, *Ee* is the eco-environment outside the system, and *Wr* is the water resources system.

The degree of economic and social development is interlaced and coupled with the natural state of the eco-environment and the availability of natural water resources. The strength of mutual influence changes with the passage of time. The fuzzy comprehensive evaluation method and entropy weight method were used to determine the efficiency of water resources, taking into account domestic, ecological, and production water usage. The outflow of water from the mainstream at different precipitation frequencies in the Mi River Basin (excluding the exchange of water between Linqu County, Qingzhou city and Shouguang city) by equation (29) was calculated based on a typical control section, and the results are shown in Table 2. In the Linqu County section of the Mihe River, the calculation of the flow from the outbound section is relatively simple because there are few tributaries. Usually, the measured inflow water from the Yeyuan Reservoir is used to subtract the economic and social water supply.

**Table 2:** Calculation results of water releases in the Mihe River Basin.

According to the monitoring value of the Mihe River Basin control section in 2019, combined with empirical formula analysis of Linqu County and Qingzhou City, the outflow water is 45 and 83 million m^3^, respectively. The water brought by typhoon transit cannot effectively replenish river ecological water, and this part of water is not considered temporarily. Based on the runoff data of the transboundary monitored sections, the runoff in Linqu County and Qingzhou City was 122 million m^3^, and the annual water flow in Yeyuan Reservoir was 80 million m^3^. Therefore, the discharge water of 128 million m^3^ in the provincial boundary section is reasonable (Fu et al., 2018, Zhang et al., 2019b).

#### 3.1.2 Spatial characteristics changes of watershed eco-compensation coupling water quantity

The ecological service value of watersheds has the characteristics of multiple dimensions, including space and time. During the study period, the ecological service value of Mihe River basin showed a relatively significant positive spatial autocorrelation and a relatively obvious spatial clustering feature (Chen et al., 2021). Scholars built eco-compensation standard model, to quantify eco-compensation amount, and obtain the watershed compensation priority on the basis of studying the temporal and spatial changes of water footprint and water surplus/deficit (Daccache et al., 2014). The incomplete mobility of water resources leads to differences in water resource utilization modes and approaches among different regions, which also forms different marginal values of water resource utilization value along with the timing changes of the implementation of ecological protection measures in the basin (Zhou, 2012). According to the characteristics of water ecosystems and the macro-operation rules of water resources, the system dynamics model of water resource value is as follows:

(30) $$S=\int_{t_{2}}^{t_{1}}F(s,\alpha ,\beta )dt$$

where *S* is the cumulative use value of water resources from $t_{1}$ to $t_{2}$ and *s* is the instantaneous use value at a certain time from $t_{1}$ to $t_{2}$, which is affected by the dual effect of water consumption growth Factor *a* and water resource decay factor *β*.

As a flowing material, water is the link in the system between the natural environment and the ecological-economic system. It is affected by the regional precipitation frequency and the stress and disturbance of the economy and society system. According to the incoming water conditions of the main stream of the Mihe River, combined with the monitored water volume of sections under different precipitation frequencies and taking into account the mutual transformation, dynamic equilibrium and coupling correlation between surface and groundwater resources, a water compensation standard for the basin is given by equation (30), with reference to the economic and social cost of water extraction in the Mihe River basin and the changes in the value of water resources (Fig. 4(b)) (Feng et al., 2021, Ysa and Nw, 2021).

When the precipitation frequency η≤50%, then:

(31) $$W=\left\{ \begin{array}{c} \left\{ \begin{array}{cc} \begin{array}{cc} (Q-0.76)\times 0.8\; & 0.41<Q<0.76\\ 0.8+(Q-0.76)\times 0.78\; & Q\geq 0.76 \end{array}\; & \text{Qingzhou City}\to \text{Linqu County} \end{array}\right.\\ \left\{ \begin{array}{cc} \begin{array}{cc} (Q-2.84)\times 0.8\; & 1.42<Q<2.84\\ 0.4+(Q-2.84)\times 0.24\; & Q\geq 2.84 \end{array}\; & \text{Shouguang City}\to \text{Linqu County} \end{array}\right. \end{array}\right.$$

When the precipitation frequency 50%<*η*≤75%, then:

(32) $$W=\left\{ \begin{array}{c} \left\{ \begin{array}{cc} \begin{array}{cc} (Q-0.41)\times 0.8\; & 0.19<Q<0.41\\ 0.8+(Q-0.41)\times 1.58\; & 0.41\leq Q<0.76 \end{array}\; & \text{Qingzhou City}\to \text{Linqu County} \end{array}\right.\\ \left\{ \begin{array}{cc} \begin{array}{cc} (Q-1.42)\times 0.8\; & 0.57<Q<1.42\\ 0.4+(Q-1.42)\times 0.49\; & 1.42\leq Q<2.84 \end{array}\; & \text{Shouguang City}\to \text{Linqu County} \end{array}\right. \end{array}\right.$$

When the precipitation frequency 75%<P≤90%, then:

(33) $$W=\left\{ \begin{array}{c} \left\{ \begin{array}{cc} \begin{array}{cc} (Q-0.19)\times 0.8\; & Q<0.19\\ 0.8+(Q-0.19)\times 3.43\; & 0.19\leq Q<0.41 \end{array}\; & \text{Qingzhou City}\to \text{Linqu County} \end{array}\right.\\ \left\{ \begin{array}{cc} \begin{array}{cc} (Q-0.57)\times 0.8\; & Q<0.57\\ 0.4+(Q-0.57)\times 1.23\; & 0.57\leq Q<1.42 \end{array}\; & \text{Shouguang City}\to \text{Linqu County} \end{array}\right. \end{array}\right.$$

Where *W* is the basin water compensation standard, US$/m^3^, and *Q* is the annual monitoring water volume of the control section under different precipitation frequencies, 100 million m^3^.

Based on the monitoring data of the control sections of the Mihe River Basin, the water compensation standards for the middle reaches of the basin in 2019 (dry year), from Qingzhou city and Shouguang city downstream to Linqu County upstream, were 0.13US$/m^3^ & 0.11US$/m^3^. The agreed amount of water released from the two sections is 41 and 57 million m^3^, and the actual amount of water released is 45 and 83 million m^3^. On the basis of comprehensive calculation and comparative analysis, the amount of water compensation from Qingzhou city and Shouguang city to Linqu County is 0.52 million US$ & 2.80 million US$, respectively. Currently, Shouguang city plans to transfer 10 million m^3^ of water from the upstream Yeyuan Reservoir. To reduce the financial transfer payment pressure of downstream Shouguang city, it is suggested to set the water price from the Yeyuan Reservoir as 0.22 US$/m^3^; after deducting the resource water price of 0.12 US$/m^3^, the ecological protection and engineering cost is only 0.10 US$/m^3^ (Mao et al., 2021; Wang et al., 2022; Zhu et al., 2022b).

#### 3.1.3 Physical properties changes of watershed eco-compensation coupling water quality

Watershed pollutants are transferred by water flow. The pollutants upstream of the basin are transported downstream through environmental media, thus affecting the water quality in the downstream reaches. To maximize the unilateral economic benefit of the basin, the reconfiguration of water resources upstream of the basin is conducive to the production of high-pollution commodities, resulting in an increase in pollutant emissions and the deterioration of water quality downstream. The “unlimited” exploitation strategy of the upstream ecological resources negatively affects the water quality downstream through socialized production and trade. The watershed protection policy includes the opportunity cost of environmental loss. However, the downstream is only willing to bear the cost of improving the water quality, to a certain extent. With the gradual increase in environmental protection costs, the industrial development list supporting the improvement of water environment quality in the basin gradually formed. The areas with good ecological endowment can realize their own development by implementing environmental protection policies and maintaining or improving the water quality of the watershed in this way.

This paper studies the pollutant flux and regional impact levels in the control section of the Mihe River Basin, which is beneficial to pollution control and ecological governance. Based on the calculation of pollutant discharge over the target water quality limit value of the control section during the research period, the pollutant compensation standard was obtained, combined with the cost of regional water pollution control. The total amount of compensation for excessive pollution is determined from a macro perspective (Dougherty et al., 2006; Peralta-Maraver et al., 2018). In the case of multiple single factors in the study period, the total compensation amount is the superposition of the compensation amount estimated by each single factor.

Based on the discharge and migration law of pollutants upstream and downstream of the watershed, the calculation formula of the watershed eco-compensation standard based on the estimation of annual pollutant flux is:

(34) $$P_{i}=W_{b,i}\times S_{i}=\int_{t_{1}}^{t_{2}}[(C_{m,i,t}-C_{o,i,t})\times Q_{t}]dt\times S_{i}$$

where $P_{i}$ is the single Factor *i* compensation standard; $W_{b,i}$ is the emission of pollutant *i* whose measured emission value exceeds the target value in the selected section period; 1) the symbol + represents the actual pollutant flux being greater than the limit value, and upstream compensates downstream; 2) the symbol - represents downstream compensation upstream; $C_{m,i,t}$ & $C_{o,i,t}$ are measured at the selected section 1 q at time *t* and the concentration of target water pollutants, respectively; $S_{i}$ is the cost of water pollution treatment per unit of contaminant *i*; and $t_{1}$ & $t_{2}$ are the starting and ending times of the study.

The *Anjialin* section on the Linqu-Qingzhou border and the *Tanfang* section on the Qingzhou-Shouguang border, which both have water quality and flow monitoring, were selected as the base sections for calculating pollutant fluxes from the four monitoring sections of the main stream of the Mihe River. The flow monitoring frequency is measured daily, and the water quality monitoring frequency is measured monthly. The water quality control target of the main stream of the Mihe River is class *v*. At this time, NH_3_-N and COD are 2.0 mg/L and 40 mg/L, respectively. The standard limit of the annual pollutant flux is calculated under the condition that the annual discharge of the *Anjialin* section and *Tanfang* section by equation (34) is 2.7 m^3^/s and 3.3 m^3^/s, respectively.

To ensure the accuracy of the calculated results, the maximum value of the calculated results is taken as the upper limit of the annual flux to form the annual flux interval (Tan et al., 2022). The compensation amount has a certain elastic interval at the upper and lower limits, which is conducive to the scientific determination of the upstream and downstream government compensation amount. The NH_3_-N and COD reduction costs of some sewage treatment plants in the Mihe River Basin are different due to different treatment processes. In this paper, the weighted calculation of pollutant reduction costs of typical enterprises in Shandong Province was combined to obtain NH_3_-N and COD unit reduction costs of 2475.42 US$/t & 640.91 US$/t. At the *Anjialin* section of the boundary between Linqu County and Qingzhou City, Linqu County needs to compensate the midstream city of Qingzhou City for exceeding the standard discharge of NH_3_-N by 31,395∼113,620 US$/t and can obtain compensation from Qingzhou City for less COD discharge by 76,395∼917,930 US$ (Table 3).

**Table 3:** Pollutants exceeding the standard of the control section in the Mihe River Basin (t/year).

where *K* is the period conversion coefficient and *n* is the number of samples.

At the junction of *Tanfang*, the pollutant emissions all meet the requirements of water function. Shouguang city in the downstream area should compensate Qingzhou city in the middle reaches for the cost of ecological and environmental improvement. The compensation intervals of NH_3_-N and COD pollutant reductions are 0.38∼0.42 million US$ and 0.62∼1.01 million US$, respectively.

The calculation formula is:

(35) $$\left\{ \begin{array}{c} W_{1}=K\sum_{i=1}^{n}\frac{C_{i}}{n}\sum_{i=1}^{n}\frac{Q_{i}}{n}\\ W_{2}=K\left(\sum_{i=1}^{n}\frac{C_{i}}{n}\right){\bar{Q}}_{r}\\ W_{3}=K\sum_{i=1}^{n}\frac{C_{i}Q_{i}}{n} \end{array}\right.\;\;\left\{ \begin{array}{c} W_{4}=K\sum_{i=1}^{n}(C_{i}{\bar{Q}}_{p}\\ W_{5}=K\frac{\sum_{i=1}^{n}C_{i}Q_{i}}{\sum_{i=1}^{n}Q_{i}}\times Q_{r} \end{array}\right.$$

To reflect the basic principles of interregional fairness and equal rights and responsibilities and fulfill the basic requirements of “whoever pollutes, compensates”, based on the optimal transfer number of pollutants in the control section of the basin, the paper presents the compensation standard based on the calculation results of the optimal pollutant reduction quota. The calculation results by equation (35) are shown in Table 4. Based on the analysis of water quality compensation standards in different situations, combined with the comparison of investment and profit in the same region, the mid-stream Qingzhou City and the downstream Shuguang City have compensated the upstream Linqu County for 1.98 million US$/year (1.98 million US$/year∼2.23 million US$/year) and 0.77 million US$/year (0.73 million US$/year∼0.80 million US$/year), respectively.

**Table 4:** Water quality compensation standards in the Mihe River Basin (Ten thousand US$/year).

Note: 1) The upstream of the *Anjialin* cross-section is Linqu County, and the downstream is Qingzhou City; 2) *Tanfang* cross-section upstream refers to Qingzhou City, and downstream refers to Shouguang City; 3) U→D means Downstream compensates Upstream, D→U means Upstream compensates Downstream.

This paper discusses the calculation method of water eco-compensation standards in cross-regional watersheds. Based on the theoretical framework of the watershed eco-compensation standard, the coupling compensation standard of water quantity and water quality is given. To realize the ecological health of the Mihe River Basin and the maximum supporting role of regional water resources for social and economic development, Linqu County, in the upstream region of the watershed, has made great sacrifices and has lost many development opportunities to improve water quality. Under the condition of ensuring a basic balance between ecological protection and socioeconomic development in the Mihe River Basin, the amount of water quantity-water quality eco-compensation from Shouguang City downstream and Qingzhou City midstream to Linqu County upstream is 4.79 million US$ and 1.28 million US$, respectively.

### 3.2 Watershed eco-compensation standard “popularization” based on bargaining & dynamic equilibrium

#### 3.2.1 Assessing the optimum value accessibility of watershed eco-compensation

This paper studies the bargaining model based on an incomplete information game. To verify the rationality of the results derived from the economic optimal strategy model, this paper uses the “perfect bargaining” and “perfect competition” modes to study the protocol characteristics generated by the perfect equilibrium and explores the applicable scope of the upstream and downstream nonzero-sum game solutions (Song et al., 2017, Xin et al., 2022).

In the face of the benefit sharing model of water resources, Linqu County upstream of the Mihe River Basin realized the balance of mixed strategies in the game of ecological protection action with the help of the bargaining model. The mixed strategy equilibrium of the complete information game is the limit of the pure strategy equilibrium of the “micro perturbation game” with incomplete information. Based on realistic research data, the cost input of ecological protection upstream of the Mihe River Basin was calculated by using the two-stage reputation game model based on Bayes' rule (Milgrom and Roberts, 1982). In period 1, both upstream and downstream of the basin participated in market competition. Upstream of the basin (“cobuilders”) take action $a_{1}$. There are two elements in the action space, that is “strive” and “compromise”. If the upstream of the basin “strive”, the downstream of the basin (“sharer”) obtains $D_{2}$, and if the upstream “compromise”, the lower reaches of the basin gain $P_{2}$, where $D_{2}>0>P_{2}$. There are two attitudes of upstream “sober” and “crazy”. The upstream of the watershed when it is sober obtains a profit of $D_{1}$ when it takes the action of “strive” and $P_{1}$ when it takes the action of “compromise”, where $D_{1}>P_{1}$. Therefore, the upstream of the watershed, with a positive attitude, would rather strive than compromise. However, from the perspective of the benefits of regional economic and social development, the revenue of each period of ecological resource consumption in the upper reaches of the basin is *M*, $M_{1}>D_{1}$. When the upstream regions of the basin are “crazy”, they take unrestrained exploitation of ecological resources, so their actions “compromise” the protection of the basin ecology. Let *p* (or 1 - *p*) represent the probability that the upstream of the watershed are sober (“crazy”).

In period 2, only the downstream basin takes action $a_{2}$. There are two types of action, including “pay” and “withdraw”. If the downstream basin chooses to pay, it receives a benefit $D_{2}$ if the upstream is “sober”, a benefit $P_{2}$ if the upstream is “crazy”, and a benefit 0 if it “withdraws”. Unless the upstream of the basin are “crazy”, it does not take a striving action in period 2; if the downstream chooses the payment attitude, the upstream of the basin will get $D_{1}$ income under sober conditions and a benefit $M_{1}$ if it “withdraws”.

Crazy watershed development behavior is considered competition for ecological resources. From a static point of view, compromising behavior in the upper basin may cause the lower basin to perceive the upper basin as “crazy” and therefore to “withdraw” ($P_{2}<0$), thus increasing the profitability of the second phase. The upstream of the basin chooses two different actions in the first phase and chooses “strive” when sober. In the separation equilibrium, the downstream basin has complete information in the second phase.

(36) $$\mu (\theta =\mathrm{sober}|a_{1}=\text{strive})=1\;\mu (\theta =\mathrm{crazy}|a_{1}=\text{compromise})=1$$

In the mixed equilibrium, the downstream basin does not update perceptions after becoming aware of the ecological compensatory equilibrium actions in the basin.

(37) $$\mu (\theta =\mathrm{crazy}|a_{1}=\text{compromise})=p$$

In a separating equilibrium, the upper basin adopts a “strive” strategy when it is sober, with a payoff of $D_{1}(1+\delta )$, where *δ* represents the discount rate between the two periods. The upstream of the basin adopts the “compromise” strategy when sober, and the lower reaches of the basin makes gains of $P_{1}+\delta M_{1}$. The necessary conditions for a separating equilibrium in the upper and lower reaches of the Mihe River Basin are as follows:

(38) $$\delta (M_{1}-D_{1})\leq D_{1}-P_{1}$$

Based on the analysis of the conditions for the establishment of separation equilibrium, the upstream watershed adopts the “strive” strategy under sober conditions. When the upper basin takes a “strive” initiative, the lower reaches of the basin assume that the upper reaches of the basin are “sober”, so they take the action of “pay”. When the “compromise” strategy is adopted in the upper reaches of the basin under the “crazy” situation, “withdraw” is chosen in the lower reaches of the basin (Yasini et al., 2015).

The costs of “compromise” are high in the upper reaches of the basin in a sober manner. If the downstream watershed “pays” in phase 2, its expected benefits for phase 2 are negative, i.e.,

(39) $$pD_{2}+(1-p)P_{2}\leq 0$$

In sobriety, the equilibrium profit upstream of the basin is $P_{1}+\delta M_{1}$, and it will gain $D_{1}(1+\delta )$ from the “strive”. Compromise is not a zero-probability event. If the “crazy” behavior is “strive” with a positive probability, then the upper reaches of the basin are “sober”.

When $D_{1}=c$ & $M_{1}=v$, the conditions for the establishment of the separation equilibrium in the first stage (c>3/4 or v<1/4) are satisfied. Similarly, the conditions for the equilibrium game in the second stage are also valid. In addition, this paper relies on the survey results of multidimensional trust willingness to pay (WTP) in the Mihe River Basin (Ni et al., 2021, Peng et al., 2021). In the upstream Linqu County of the Mihe River Basin, the monthly investment cost of “strive” in the “sober” state was 0.52 US$/person. In the middle and lower reaches of the basin, the ecological benefit value of “payment” is 1.40 US$/person under the influence of the “sober” action of the upper reaches. Based on the nonzero-sum treatment of the survey results, the current relationship between the value of ecological compensation inputs and the willingness to pay for ecological benefits in the watershed satisfies v≥c+1/4. Therefore, it is reasonable for downstream Shouguang City and middle Qingzhou City to calculate water quantity and quality eco-compensation quotas of 4.78 million US$ and 1.29 million US$, respectively, for upstream Linqu County. This provides a scientific basis for ecological protection and sustainable development of the basin (Liu et al., 2021b).

#### 3.2.2 Realizing the popularization of watershed eco-compensation based on data statistical analysis

Economically valuing the non-monetary ecosystem services often proves difficult, rendering revealed preference methods inapplicable. We conducted a discrete decision experiment to elicit the preferences and WTP of the watershed ecosystem services in the Mihe River Basin, make strong quantifying support for watershed eco-compensation standard “Popularization”. The respondents' groups were divided according to the industrial layout, population composition, public awareness of ecological protection and regional ecological protection objectives of the Mihe River basin. The attribute characteristics of the sample are shown in Table 5. The stratified sampling procedure was followed to obtain a representative non-zero-sum sample. Given this and that several uncooperative respondents were removed, the sample does differ slightly from the population of Weifang City (Fig. 3). The ecological protection of the respondents as well as the attitudes, social norms and perceptions behavior control towards the payment for sustainable integrated management were analyzed through a series of items (Table 5), the Cronbach's alpha is α=0.41 (Johnson and Geisendorf, 2022). Table 5 reports the overall mean score and standard deviations for different groups of respondents. A Pearson correlation test revealed significant positive correlations (p<0.001) between all variable's perceptions behavior control and ecological protection consciousness. The number of samples can meet the evaluation requirements, and the sample statistical method is scientific and reasonable (Darío et al., 2018, Dang et al., 2021).

**Table 5:** Data statistical characteristics of the investigation sample.

The conditional logit model and class models were used to estimate the eco-compensation Optimized results. We estimated three models, each with a different set of variables interacting with the watershed eco-compensation (WEC) variable (Sarrias et al., 2018). Model 1 is consisting of WEC & ATW, model 2 is made up of WEC, SN, and PBC, and model 3 is composed of WEC, ATW, SN, PBC, NEPP, as well as watershed variation characteristics. Based on the criteria AIC (Akaike Information Criterion) and BIC (Bayesian Information Criterion), optimal model is used to calculate additional interaction variables. In order to estimate the willing to pay for watershed eco-compensation, we calculated the mean marginal rates of substitution of the cost parameter for each respective group. Results for the three conditional logit models are given in Table 6.

**Table 6:** Quantification results of watershed eco-compensation based on data statistical models.

Attribute value list	Model 1		Model 2		Model 3		Model 1(US$/month)		Model 2(US$/month)		Model 3(US$/month)	
	Coefficient	Standard error	Coefficient	Standard error	Coefficient	Standard error	WTP	Standard error	WTP	Standard error	WTP	Standard error
WEC	0.100	0.078	0.117	0.095	−0.011	0.102	3.02	1.990	3.53	2.329	−0.29	2.343
HEAT2	0.102^##^	0.047	0.102^##^	0.047	0.102^##^	0.049	3.10^##^	1.213	3.04^##^	1.209	2.92^##^	1.155
HEAT3	0.254^###^	0.048	0.258^###^	0.048	0.269^###^	0.048	7.69^###^	1.274	7.67^###^	1.266	50.87^###^	1.209
WATER2	0.524^###^	0.051	0.528^###^	0.051	0.541^###^	0.051	15.87^###^	1.580	15.84^###^	1.573	7.61^###^	1.487
WATER3	0.805^###^	0.050	0.807^###^	0.050	0.822^###^	0.050	24.33^###^	2.037	24.21^###^	2.022	23.35^###^	1.899
DIV2	0.350^###^	0.049	0.352^###^	0.049	0.356^###^	0.051	10.57^###^	1.469	10.50^###^	1.459	10.10^###^	1.383
DIV3	0.452^###^	0.047	0.449^###^	0.047	0.465^###^	0.048	13.54^###^	1.509	13.47^###^	1.499	13.14^###^	1.424
AES2	0.409^###^	0.053	0.412^###^	0.053	0.423^###^	0.004	12.34^###^	1.466	12.31^###^	1.465	12.02^###^	1.383
AES3	0.558^###^	0.049	0.551^###^	0.049	0.554^###^	0.061	16.50^###^	1.602	16.52^###^	1.598	15.74^###^	1.985
COST	−0.042^###^	0.005	−0.042^###^	0.005	−0.042^###^	0.085						
*AGE*			0.340^###^	0.056	0.279^###^	0.086			10.19^###^	1.516	7.89^###^	1.497
*GENDER*			−0.012	0.079	−0.088	0.061			−0.39	1.870	−2.51	1.504
*INCOME*			−0.179^##^	0.082	−0.075	0.076			−5.36^##^	1.969	−2.12	1.939
*EDUCATION*			−0.119	0.080	−0.075	0.063			−3.55	1.943	−2.10	1.995
*ATW*					−0.507^###^	0.062					−14.36^###^	1.701
*SN*					−0.582^###^	0.076					−16.48^###^	2.053
*PBC*					−0.436^###^	0.061					−12.32^###^	1.653
*NEPP*					−0.503^###^	0.063					−14.30^###^	1.746
*SWCHARGE*					0.561^###^	0.106					15.94^###^	2.664
Log-likelihood-null	−4697.860		−4697.860		−4697.860							
Log-likelihood	−4375.550		−4375.550		−4062.190							
AIC	8776.100		8738.090		8165.360							
BIC	8840.160		8826.860		8285.120							
Observations	4480.000		4480.000		4480.000							

Note: (1) Significance level, ^###^p<0.01, ^##^p<0.05, ^#^p<0.1; (2) *AGE*, Italics represent variables that interact with the WEC.

After fitting the Logit model coefficients, considering the monetary attribute of eco-compensation cost, the marginal WTP of a certain attribute level can be calculated by dividing the attribute coefficient by the monetary attribute coefficient (Hoyos, 2010). According to the attribute parameters given by the discrete choice experiment of the questionnaire, the compensating surplus (CS) was calculated according to Hanemann (1984):

(40) $$CS=-\frac{1}{\alpha }(\ln\sum e^{V_{1}}-\ln\sum e^{V_{0}})$$

Where *α* is the monetary attribute coefficient representing the marginal utility of income, and $V_{0}$ & $V_{1}$ are the indirect utility functions of the state before and after the change, respectively.

The marginal willingness to pay for eco-compensation in the Mihe River Basin is closely related to the respondents' ability to pay, the change of water resource endowments, and the regional temperature level. The result of conditional Logit model is an optimal result based on the factors such as potential willingness to pay, paying consciousness of interviewees, consumer surplus (CS), combining capacity between NbS and social system. In the case of optimal allocation of social resources, the willingness to pay in the Mihe River Basin is 65.63 million US$/month by equation (40) (Table 7). The discrete choice experiment shows that payment preference and payment willingness are very important in the implementation of watershed eco-compensation standards. Respondents with strong environmental protection awareness are willing to pay a lot of money to increase the implementation effectiveness of ecological conservation. In addition, residents with high scores in attitude, social norms and perceptions behavior control were also more willing to pay for eco-compensation. With the help of cost-benefit analysis, the optimized eco-compensation standard has a strong popularity. Watershed eco-compensation standard based on NbS is shown in the Fig. 5.

**Table 7:** The marginal WTP optimal value calculated with conditional Logit models.

Attribute value list	Reference		Low WTP		Water WTP		High WTP		No WTP		No WTP^**a**^
	(US$/month)		(US$/month)		(US$/month)		(US$/month)		(US$/month)		(US$/month)
	WTP	Standard	WTP	Standard	WTP	Standard	WTP	Standard	WTP	Standard	Average
		error		error		error		error		error	
WEC	7.59^##^	2.437	−2.08^##^	0.785	−42.39^###^	12.500	−71.86^###^	17.280	−13.39	17.279	−44.24
HEAT2	−0.09	1.987	1.54^#^	0.652	2.20	3.776	5.09	2.570	23.64	2.572	3.23
HEAT3	−1.17	1.950	1.52^#^	0.709	7.42	4.536	13.62^###^	3.356	26.41	3.350	8.46
WATER2	0.85	1.952	1.26	0.658	12.00^#^	5.022	30.34^###^	5.594	5.15	5.594	17.62
WATER3	1.31	1.708	1.96^##^	0.689	12.27^##^	4.911	46.43^###^	8.728	6.22	8.729	25.47
DIV2	−0.19	2.290	0.87	0.778	3.53	3.660	19.30^###^	4.590	12.21	5.586	10.16
DIV3	2.00	2.382	2.05^#^	0.863	3.31	3.726	24.38^###^	5.022	35.92	5.022	12.88
AES2	−0.88	2.034	1.57	0.978	8.84^#^	4.142	26.05^###^	4.798	−10.57	4.798	14.73
AES3	0.76	1.965	2.67^###^	0.828	1.53	3.800	34.59^###^	6.796	17.19	6.798	17.32

Note: (1) Significance level, ^###^p<0.01, ^##^p<0.05, ^#^p<0.1; (2) a, average WTP weighted by the share within classes excluding the NO WTP.

**Figure 5:** Interactive influences of ecosystem services and socioeconomic factors on watershed eco-compensation standard “popularization” in the quantifying process of bargaining & dynamic equilibrium. The figure presents the calculation process of watershed eco-compensation standards oriented to economic optima and equilibrium games based on NbS, which expands the current calculation thought in this area.

## 4 Results discussion

### 4.1 Existence of the bargaining optimization solution

In most models, classical Pareto optimality can be achieved through participants' behavior deviating from the equilibrium (Audet et al., 2022). In the process of determining the watershed ecological compensation standard based on bargaining, if the upstream and downstream of the watershed can communicate effectively, from the perspective of balanced transactions, the two sides can form an efficient transaction mechanism. Under the current incentive compatibility mechanism, the significance of efficiency lies in the maximization of overall benefits upstream and downstream of the basin. There is an efficient incentive compatibility mechanism (g,x) if, and only if, there is no other incentive compatibility mechanism ($\overset{ˆ}{g},\overset{ˆ}{x}$), such that for every $v_{1}$ and $v_{2}$ between 0 and 1, then

(41) $$\left\{ \begin{array}{c} U_{1}(v_{1},\overset{ˆ}{g},\overset{ˆ}{x})>U_{1}(v_{1},g,x)\\ U_{2}(v_{2},\overset{ˆ}{g},\overset{ˆ}{x})>U_{2}(v_{2},g,x) \end{array}\right.$$

Relying on the research of Holmström and Myerson (1983), the above concept of efficiency is equivalent to the weakened form of interim incentive efficiency. A bargaining analysis of the equilibrium solution of the watershed eco-compensation standard is carried out to ensure the effective implementation of the watershed eco-compensation standard. In this paper, three mechanisms proposed by Chatterjee and Samuelson (1983) are used to explore the theoretical rationality of equilibrium solution results.

① The upstream seller has the right to demand any price for his subject matter, and the downstream buyer may accept or reject the criterion. During the game, the seller's optimal price is $q_{1}=(1+{\overset{˜}{V}}_{1})/2$, and the expected profit maximization of the price is $\left(1-q_{1})(q_{1}-V_{1}\right)$. Therefore, this mechanism can be expressed as, ($g^{1},x^{1}$), where:

(42) $$\left\{ \begin{array}{c} g^{1}(v_{1},v_{2})=\left\{ \begin{array}{cc} 1\; & v_{2}\geq \frac{1+v_{1}}{2}\\ 0\; & v_{2}<\frac{1+v_{1}}{2} \end{array}\right.\\ x^{1}(v_{1},v_{2})=\left\{ \begin{array}{cc} \frac{1+v_{1}}{2}\; & v_{2}\geq \frac{1+v_{1}}{2}\\ 0\; & v_{2}<\frac{1+v_{1}}{2} \end{array}\right. \end{array}\right.$$

Based on the findings of Holmström and Myerson (1983), ($g^{1},x^{1}$) is effective.

(43) $$\left\{ \begin{array}{c} L_{1}(v_{1})=v_{1}\\ L_{1}(v_{2})=\left\{ \begin{array}{cc} 0\; & v_{2}=0\\ 1\; & v_{2}>0 \end{array}\right. \end{array}\right.$$

Combined with the analysis, the trading area of the mechanism ($g^{1},x^{1}$) is shown in Fig. 6(a).

**Figure 6:** The integrated approach based on NbS in achieving sustainability of socio-economic & ecosystem management. It can promote the synergy of multiple multilateral environmental agreements. Harness watershed eco-compensation toward basin-level ecological-economic-social synergy objectives. The setting of equilibrium points, developed through basin-wide dynamic Bayesian game, coupling and coordination analysis and subsequent basin management plans, would provide valuable guidance for subnational programs, and help largest ecosystem synergies tradeoffs. Build coordination and consultation mechanisms among different participants which can help watershed eco-compensation programs be more effective, efficient, and equitable.

② The downstream buyer can commit to any offer for the subject matter, and then the seller can only accept or reject the offer. In this game, the buyer's optimal price is $q_{2}=(1+{\overset{˜}{V}}_{2})/2$, and the expected profit maximization of the price is $q_{2}({\overset{˜}{V}}_{2}-q_{2})$. Therefore, this mechanism can be expressed as, ($g^{2},x^{2}$), where:

(44) $$\left\{ \begin{array}{c} g^{2}(v_{1},v_{2})=\left\{ \begin{array}{cc} 1\; & \frac{v_{2}}{2}\geq v_{1}\\ 0\; & \frac{v_{2}}{2}<v_{1} \end{array}\right.\\ x^{2}(v_{1},v_{2})=\left\{ \begin{array}{cc} \frac{v_{2}}{2}\; & \frac{v_{2}}{2}\geq v_{1}\\ 0\; & \frac{v_{2}}{2}<v_{1} \end{array}\right. \end{array}\right.$$

The mechanism ($g^{2}$, $x^{2}$) is efficient, and the trading area is shown in Fig. 6(b).

③ The upstream and downstream regions of the watershed at the same time. If the upstream seller's offer in the basin is lower than the downstream buyer's offer, then the buyer is compensated according to the average of the two offers. If the seller's price is higher than the buyer's, the transaction is broken. Chatterjee and Samuelson (1983) show that the equilibrium price of the game is $q_{1}=\frac{2}{3}{\overset{˜}{V}}_{1}+\frac{1}{4}$, $q_{2}=\frac{2}{3}{\overset{˜}{V}}_{2}+\frac{1}{12}$. It holds at $q_{1}\geq q_{2}$, when and only when ${\overset{˜}{V}}_{2}\geq {\overset{˜}{V}}_{1}+\frac{1}{4}$. Therefore, this mechanism can be expressed as ($g^{3},x^{3}$), where:

(45) $$\left\{ \begin{array}{c} g^{3}(v_{1},v_{2})=\left\{ \begin{array}{cc} 1\; & v_{2}\geq v_{1}+\frac{1}{4}\\ 0\; & v_{2}<v_{1}+\frac{1}{4} \end{array}\right.\\ x^{3}(v_{1},v_{2})=\left\{ \begin{array}{cc} \frac{v1+v_{2}+\frac{1}{2}}{3}\; & v_{2}\geq v_{1}+\frac{1}{4}\\ 0\; & v_{2}<v_{1}+\frac{1}{4} \end{array}\right. \end{array}\right.$$

The mechanism ($g^{3}$, $x^{3}$) is efficient, and the trading area is shown in Fig. 6(c).

In the above three feasible mechanisms, ($g^{3}$, $x^{3}$) maximizes the sum of the expected profits of the two traders, i.e.,

(46) $$\left\{ \begin{array}{c} L_{1}(v_{1})=\left\{ \begin{array}{cc} \frac{2v_{1}}{3}\; & v_{1}<1\\ 1\; & v_{1}=1 \end{array}\right.\;L_{2}(v_{2})=\left\{ \begin{array}{cc} 0\; & v_{2}=0\\ \frac{2v_{2}}{3}+\frac{1}{3}\; & v_{1}<0 \end{array}\right.\\ \int_{0}^{1}U_{1}(v_{1},g,x)dL_{1}(v_{1})\int_{0}^{1}U_{2}(v_{2},g,x)dL_{2}(v_{2})=\frac{2}{3}[\int_{0}^{1}U_{1}(v_{1},g,x)dv_{1}+\int_{0}^{1}U_{2}(v_{2},g,x)dv_{2}+\frac{1}{2}U_{1}(1,g,x)+\frac{1}{2}U_{2}(0,g,x)] \end{array}\right.$$

The expression in square brackets is the Lagrange function of the maximization of expected total profit upstream and downstream of the watershed when a 1/2 shadow price is assigned to individual rational constraints $U_{1}(1,g,x)\geq 0$ & $U_{2}(0,g,x)\geq 0$. The above three incentive compatibility mechanisms, ($g^{3},x^{3}$) can maximize the individual benefits of participants and make the equal sign of individual rational constraints upstream and downstream of the basin valid. Therefore, all feasible mechanisms, ($g^{3},x^{3}$) can maximize the expected total profits of eco-compensation in the basin. The discussion shows that the proposed method can be used to deal with the redundant information in the game process to facilitate bargaining and obtain the optimal solution of the dynamic game process. Of course, the possibility of information acquisition modeling research is very specific work, and the paper focuses on the application of general methods. When the upstream and downstream of the basin are asymmetric on eco-compensation standards, the influence of the parties' reputation and the existence of third-party arbitration have an important impact on the solution of the balanced solution of compensation standards.

### 4.2 Efficiency of the watershed eco-compensation standard

Equilibrium solutions of incomplete information games are not all inefficient. The inefficiency of the bargaining game deviates somewhat from the findings of Bhattacharya (1982) for the case of free competition. If only incomplete information is provided unilaterally downstream of the basin and if the value of ecological services in the basin is variable, then it is easy to develop an efficient mechanism based on a complete information game. The concept of implementation efficiency of watershed ecological compensation is difficult to define in incomplete information games. In the bargaining game, upstream and downstream participants of the basin try to reach agreement on the model to be used in the actual bargaining. Once the pattern is adopted, participants can solve actual bargaining “free-for-all” problems by implementing balanced strategies. For participants upstream of the basin, even though the downstream of the basin tends to implement eco-compensation, the “free-for-all” model is no longer incentive compatible. Watershed participants expect to receive nonnegative compensation before the compensation standard is formed. The probability distribution of watershed willingness to pay is continuous and positive in their respective domains. Therefore, complete information efficiency and individual rationality are incompatible in the game process.

Before the formation of the watershed eco-compensation standard, the payment behavior of upstream and downstream participants was individual rational. Since the price of individual willing payments is distributed independently, the eco-compensation standard based on a complete information game is efficient in the case of unilateral payments by watershed participants (D'Aspremont and Gerard-Varet, 1979; Chatterjee, 1982). If there is “crazy” irrational action in the upstream and downstream of the basin, the participants play the game to maximize unilateral benefits, and then the winner then expects to receive a lump sum of compensation that is not subject to bargaining. Therefore, under the constraints of incentive compatibility and individual rationality, Chatterjee and Samuelson (1983) showed that the expected eco-compensation amount of upstream and downstream watersheds could be maximized by game (subject to uniform distribution [0,1]). To maximize the expected value of the ecological compensation standard, there is no other incentive compatible mode for the upstream and downstream participants under the premise of the “incentive efficiency” mechanism. The optimal model maximizes the “substantial utility” of participants. “Substantial utility” is the cost required after subtracting the actual utility from the incentive compatibility constraint, which is the “neutral bargaining mechanism” satisfying the Nash axiom.

The upstream and downstream participants negotiate on the choice of ecological compensation model. In noncooperative games, to satisfy the constraints of information availability and the corresponding mechanism requirements, the strategy choice of participants cannot be given by any unilateral party under the consideration of incentive compatibility. The participants can form enforceable opinions before the game starts, limiting the outcome of the game to the desired objective. Disobedience can be detected and should be punished. Participants can be “coerced” into forming bargaining strategies through “closed” discussions before the expected compensation standards are known upstream and downstream of the basin. The noncooperative game requires that the watershed participants make decisions and abide by them, and the bargaining behavior is limited to the category of “policy optimization”. The “closed” negotiation cannot achieve the perfect equilibrium of the reasonably designed bargaining game. Watershed eco-compensation standards are implemented dynamically in stages. Balance is perfect during the implementation of the order stage. The implementation result of the bargaining mechanism provides technical support for the expected payment amount and the implementation time of the compensation standard. In the equilibrium of an incomplete information game, the possibility of delayed agreement inefficiency is low.

Based on the research results of scholars, the calculation results will be more equitable for upstream and downstream compensation. Taking the Taihu Basin as an example, based on the econometric loss calculation model, Zhenjiang City's compensation for local and downstream areas was 1.021 billion yuan, the watershed eco-compensation standard is determined mainly by the water pollution economic loss (Lu et al., 2020). We obtained watershed eco-compensation via practices based on the actual situation. China is one of the largest polluters in the world, to analyze transboundary pollution control options between a compensating and compensated region, a stochastic differential game model to determine and contrast outcomes across both cooperative and non-cooperative game scenarios (Jiang et al., 2019b). To achieve the benefits of ecological protection, combining gross ecosystem product accounting with total cost accounting could pose huge economic pressure on payers. Based on basin eco-compensation standard valuation for cross-regional water supply, water-related ecosystem services received a minor proportion (<3%) of the compensation (Fang et al., 2021). To construct a long-term and sustainable watershed eco-compensation mechanism for the protection of water resources and sustainable development, local governments and polluting enterprises should participate together. The increase of marginal decline degree of value function will lead to a significant reduction in the time for the local governments to reach a stable state (Shen et al., 2021). Therefore, the central government should minimize the possibility of the downstream government's non-commitment. In addition, compared with the research results of Huang et al. (2010), the research results are scientific and reliable, which confirms the rationality of the values in this paper.

The discrete choice experiment shows that payment preference and payment willingness are very important in the implementation of watershed eco-compensation standards. Respondents with strong environmental protection awareness are willing to pay a lot of money to increase the implementation effectiveness of ecological conservation. In addition, residents with high scores in attitude, social norms and perceptions behavior control were also more willing to pay for eco-compensation. With the help of cost-benefit analysis, the optimized eco-compensation standard has a strong popularity. During multistage watershed eco-compensation standard implementation, due to the complexity of practical problems, there may be unbalanced behavior, but the inefficiency caused by incomplete information is not as serious as expected by theoretical game behavior. The implementation conditions, implementation process and implementation effect of eco-compensation in the Mihe River Basin are based on rational requirements and comprehensive analysis in the process of balanced game realization, which is the comprehensive analysis result with efficiency. In a follow-up study, the efficiency of the implementation of watershed ecological compensation will be considered in the category of information economics or uncertain economics, and the general inefficiency caused by incomplete information and different environments will be accurately solved.

## 5 Conclusions

The research method presented in this paper is suitable for studying the coordination relationship between the upstream and downstream river basins and ecological protection. This paper establishes the multivariate equilibrium game model of uncertain information to dynamically determine the watershed eco-compensation standard, determines the rationality of the compensation standard result through bargaining, and explores the watershed eco-compensation standard measurement system based on economic optimization analysis.

In combination with the economic and social water drawing cost standard and the changing law of water resource use value in the Mi River Basin, from the perspective of water ecological value, the compensation amount of water volume from Qingzhou City in the middle reaches and Shouguang City in the lower reaches to Linqu County in the upper reaches is 0.52 million US$ & 2.80 million US$, respectively. Based on the optimal transfer amount of pollutants in the control section of the watershed, this paper calculates the water quality compensation standard based on the optimal reduction quota of pollutants. In the analysis of water quality compensation standards in different situations, combined with the same regional investment and profit quota, the water quality compensation quota of Qingzhou City in the middle stream and Shouguang City in upstream Linqu County was 0.77 million US$/year and 1.98 million US$/year, respectively. In ensuring the basic balance between ecological protection and social and economic development in the Mi River basin, downstream Shouguang City and midstream Qingzhou City have offered ecological compensation quotas of 4.78 million US$ and 1.29 million US$, respectively, for upstream Linqu County. Based on the nonzero-sum processing of the survey results, the current relationship between the input value of ecological compensation and the willingness to pay satisfies v≥c+1/4. Based on the dynamic game & Bayesian equilibrium solution of bargaining, the watershed eco-compensation quota of water quantity & quality is 6.07 million US$, the willingness to pay is 65.63 US$/month.

Combining capacity between NbS and social system, the result of conditional Logit model is an optimal result. The research method presented in this paper can be used to deal with the redundant information in the process of the game to facilitate bargaining and obtain the optimal solution of the dynamic game process. The research results of this manuscript are conducive to optimizing the construction mode of watershed horizontal eco-compensation and improving the compensation path of market diversification. In subsequent studies, the optimization of equilibrium solutions and the efficiency of implementation of eco-compensation in watersheds will be considered in the context of information or uncertain economics, taking into account the subjective thinking of the participants, to address the complex issues that constrain the efficiency of eco-compensation implementation.

## Declarations

### Author contribution statement

**Yicheng Fu; Wenqi Peng:** Conceived and designed the experiments; Wrote the paper.

**Jinyong Zhao; Gensheng Fu:** Performed the experiments; Wrote the paper.

**Yicheng Fu; Jian Zhang:** Analyzed and interpreted the data; Wrote the paper.

**Jian Zhang; Gensheng Fu:** Contributed materials and analysis data; Wrote the paper.

### Funding statement

Professor Yicheng Fu was supported by 10.13039/501100011395Major Science and Technology Program for Water Pollution Control and Treatment [2018ZX07105002]. Jian zhang was supported by 10.13039/501100012165Key Technologies Research and Development Program [2016YFC0401408].

### Data availability statement

Data included in article/supp. material/referenced in article.

### Declaration of interests statement

The authors declare no competing interests.

### Additional information

No additional information is available for this paper.
